The article "Comprehensive Analysis of Subtypes and Identification of Key lncRNAs Based on Glutamine Metabolism-Related Long Noncoding RNAs" was retracted in 2023. Reasons: signs of a paper mill; compromised peer review; unreliable results or conclusions.

# Comprehensive Analysis of Subtypes and Identification of Key lncRNAs Based on Glutamine Metabolism-Related Long Noncoding RNAs

**DOI:** 10.1155/2022/2807354

**Published:** 2022-04-29

**Authors:** Yuwei Feng, Xiaowei Sun, Tiangu Yang, Jingqi Han, Dapeng Zhou, Haitao Ren, Yulong Sheng, Yanhua Wang

**Affiliations:** ^1^Department of Interventional Medicine, Affiliated Hospital of Qingdao University, No. 16, Jiangsu Road, Shinan District, Qingdao, Shandong Province, China; ^2^Department of Medical Imaging, Qingdao Women and Children's Hospital, 6 Tongfu Road, Shibei District, Qingdao, Shandong, China; ^3^Department of Interventional Medicine, Affiliated Hospital of Qingdao University, 369 Shanghai Road, Pingdu, Qingdao, Shandong, China

## Abstract

**Background:**

Long noncoding RNAs (lncRNAs) are becoming a critical class of metabolic regulate molecule in cancer. Glutamine is a regulator that contributes to each of the core metabolic tasks in proliferating tumor cells. Thus, we aimed to evaluate the association of lncRNAs with glutamine metabolism in lung adenocarcinoma (LUAD).

**Methods:**

Using single-sample gene set enrichment analysis (ssGSEA), LUAD specimens were assigned scores based on glutamine metabolism-related genes, and the shared common glutamine metabolism-related lncRNAs in three different LUAD data cohorts were identified. ConsensusClusterPlus was used to perform unsupervised clustering analysis in patients with LUAD. Key glutamine metabolism-related lncRNAs were identified by first-order partial correlation analysis.

**Results:**

A total of 11 shared glutamine metabolism-associated lncRNAs were identified in three LUAD data cohorts, and LUAD patients were classified into three glutamine metabolism subtypes based on the expressions of the related genes. C1 exhibited shorter overall survival (OS), poor genomic instability, and inadequate infiltration of immune cell types in the tumor microenvironment (TME) and was representative of the immunodeficiency phenotype. C2 represented the immunosuppressive phenotype while C3 represented the immune activation phenotype, exhibiting the highest sensitivity to immunotherapy. Nine of the 11 lncRNAs were localized to the nucleus. Finally, three key lncRNAs, significantly enriched in multiple metabolic pathways, were screened and found to be remarkably related to the OS of LUAD.

**Conclusion:**

We identified three glutamine metabolism subtypes of LUAD, which reflected different OS, genomic, and TME features, and identified three key glutamine metabolism-associated lncRNAs may contribute to further study of lncRNAs in cancer metabolism.

## 1. Introduction

Glutamine has traditionally been considered a nonessential amino acid and is a vital source of nitrogen and carbon for cellular processes involving biosynthesis. Glutamine is synthesized by most mammalian tissues; however, owing to their rapid proliferation and growth, cancer cells exert a strong demand for glutamine [1]. The main reason attributed for this need in proliferating tumor cells is that glutamine essentially contributes to each core metabolic process as follows: it supports cellular defense against oxidative stress, is involved in bioenergetics, and supplements glucose metabolism for the synthesis of other macromolecules [2]. Moreover, in some cancer cells, in exchange for leucine and other essential amino acids, glutamine is exported, which regulates cell growth, protein translation, mTOR stimulation, and autophagy through serine/threonine kinases [3]. Those features make glutamine metabolism a putative target for the development of novel clinical regimens for the detection, monitoring, and treatment of cancer [4].

The article "Comprehensive Analysis of Subtypes and Identification of Key lncRNAs Based on Glutamine Metabolism-Related Long Noncoding RNAs" was retracted in 2023. Reasons: signs of a paper mill; compromised peer review; unreliable results or conclusions.

Recent advances in the transcriptomic analysis of noncoding RNAs have led to the identification of the regulatory processes of glutamine metabolism in oncocytes. The miR-145 in ovarian carcinoma by targeting c-myc/Glutaminase-1 (GLS1) suppresses glutamine metabolism in cancer cells [ 5]. MiR-9-5p regulates the expression of glutamic-oxaloacetic transaminase 1 (GOT1) in pancreatic carcinoma, hence impeding glutamine metabolism and redox homeostasis [6]. Circ-MBOAT2, showing an aberrantly high expression in pancreas carcinoma tissues and cells, regulates glutamine catabolism and tumor progression through the miR-433-3p/GOT1 signaling axis [7]. lncRNA by definition is a transcript longer than 200 nucleotides. They have been reported to regulate tumor glutamine metabolism through different mechanisms. lncRNA EPB41L4A-AS1 modulates glycolysis and glutamine catabolism via the mediation of the nucleolar translocation of histone deacetylase-2 (HDAC2) [8]. lncRNA UCA1 enhances glutamine metabolism in human bladder cancer cells by targeting miR-16 [9]. The OIP5-AS1 sponge adsorbs miR-217 to upregulate the expressing of glutaminase (GLS), hence facilitating tumor proliferation and glutamine catabolism in melanoma [10]. Therefore, lncRNAs are regulators of glutamine metabolism, and comprehensive analysis of the tumor transcriptome from the perspective of glutamine metabolism-related lncRNAs is a potential strategy to reveal the causal links beneath tumor metabolism.

Herein, a total of 1097 samples were collected from three independent LUAD cohorts and from which lncRNA and mRNA expression profiles were extracted. The glutamine metabolism-related lncRNAs were screened, and glutamine metabolism subtypes were identified based on their expression in the LUAD samples. Next, we examined the characteristics of glutamine-metabolizing subtypes for genomic alterations, TME, and immunotherapeutic response. Finally, potential regulatory pathways of glutamine metabolism-related lncRNAs were evaluated, and key lncRNAs affecting the LUAD prognosis were identified.

The article "Comprehensive Analysis of Subtypes and Identification of Key lncRNAs Based on Glutamine Metabolism-Related Long Noncoding RNAs" was retracted in 2023. Reasons: signs of a paper mill; compromised peer review; unreliable results or conclusions.

## 2. Materials and Methods

### 2.1. Transcriptome Dataset for LUAD

The RNA-seq data and relevant prognostic data for LUAD samples were retrieved from TCGA and GEO (accession numbers GSE31210 [11] and GSE72094 [12]) databases. Of these, 485 LUAD samples were extracted from TCGA, and 226 and 386 LUAD samples were extracted from GSE31210 and GSE72094, respectively. To obtain the lncRNA expression profiles from the two cohorts of the GEO database, we first separately downloaded the fasta files for the probe sequence corresponding to their microarray platforms and entered them into the GENCODE website [13] (https://www.gencodegenes.org/human/) to download the latest version of the corresponding transcriptome reference sequence fasta file (GRCh38.p13). Next, the sequence of the probe was compared with the transcriptome fasta sequence using SeqMap [14] with the number of mismatches set to 0 for obtaining the new probe annotation file. Finally, the latest GTF file was also downloaded from the GENCODE website (https://ftp.ebi.ac.uk/pub/databases/gencode/Gencode_human/release_39/gencode.v39.annotation.gff3.gz), and the microarray data were divided into mRNAs and lncRNAs according to the annotations in the file. Figure S1 shows the whole workflow of this study.

### 2.2. Identification of Glutamine Metabolism-Related lncRNAs

The glutamine metabolism-related genes belonging to the GOBP GLUTAMINE FAMILY AMINO ACID METABOLIC PROCES gene set were obtained from the MSigDB [15] (HTTPS://http://www.gsea-msigdb.org/). Using GSVA [16] in the R software, the ssGSEA was performed, and glutamine metabolism scores were computed for every specimen in TCGA, GSE31210, and GSE72094 cohorts. Pearson correlation coefficient with a threshold of ∣cor | >0.3 and *P* < 0.05 was set to identify the glutamine metabolism-related lncRNAs.

### 2.3. Cluster Analysis for Patients with LUAD

The extracted glutamine metabolism score-related lncRNAs were input for unsupervised clustering analysis using the partitioning around medoid clustering (PAM) algorithm. This step was performed using the R package, ConsensusClusterPlus [17]. The clustering parameters were set as follows: *k* = 2-10, bootstraps = 500, and pItem = 0.8. The optimum number of clusters was identified using the CDF curves.

### 2.4. Mutation Analysis

We calculated the aneuploidy score, homologous recombination defects (HRDs), fraction altered, number of segments, and tumor mutation burden (TMB) to compare the obtained genomic stability in different clusters. Using the GenVisR [18] R package, genetic mutations and copy number variants were compared among the clusters, and the top 10 most significantly mutated genes, copy number amplifications, and deletions were presented using a Waterfall plot.

The article "Comprehensive Analysis of Subtypes and Identification of Key lncRNAs Based on Glutamine Metabolism-Related Long Noncoding RNAs" was retracted in 2023. Reasons: signs of a paper mill; compromised peer review; unreliable results or conclusions.

### 2.5. Gene Set Enrichment Analysis (GSEA) with Functional Annotation

The gene sets from the Hallmark database [15] were used as a “list of reference genes” for GSEA. The R package [19], clusterProfiler [20] (https://guangchuangyu.github.io/software/clusterProfiler), was used for functional annotation, and the enrichment of different pathways in each cluster was obtained, where false discovery rate (FDR) < 0.05 represented significant enrichment.

### 2.6. Analysis of Immune and Stromal Infiltration

The marker genes for all immunocytes were acquired from Senbabaoglu et al. [21]. Using ssGSEA, the enrichment scores were calculated, which represented the relative abundance of immunocytes in each sample in its TME. The Estimation of STromal and Immune cells in MAlignant Tumours using Expression algorithm (ESTIMATE; https://sourceforge.net/projects/estimateproject/) was employed to compute the stromal and immunoscores and assess the differences in TME components among the different clusters.

### 2.7. Response Prediction for Immunotherapy

The information on immune checkpoints was obtained from the HisgAtlas database [22] to analyze whether they were differentially expressed among the clusters. Because of insufficient publicly available data in LUAD cohorts receiving immune therapy, our team utilized the TIDE [23] arithmetic to preliminarily examine the responsiveness of patients in different cohorts to immune checkpoint blockade (ICB).

### 2.8. Analysis of Transcription Factor Activity

The transcription factor (TF) activity was scored for each sample as per the approach proposed by Garcia-Alonso et al. [24]. Using analysis of variance (ANOVA), the TF activation levels were compared among the clusters, and *P* < 0.05 was used as a screening criterion to identify the TFs that showed significant differences.

### 2.9. Identification of Key Glutamine Metabolism-Associated lncRNAs by First-Order Partial Correlation Analysis

The first-order partial correlation analysis was completed to investigate the association between lncRNAs and glutamine metabolism-related genes. Glutamine metabolic fraction was considered as *x* and glutamine metabolism-associated genetic expression as *y*. The following was the computation for the first-order partial correlation between *x* and *y* for lncRNAs:

(1) $$\begin{array}{c} r_{xy\text{lncRNA}}=\frac{rxy-rx\text{lncRNA}*ry\text{lncRNA}}{\sqrt{\left(1-r_{x\text{lncRNA}}^{2}\right)}*\left(1-r_{y\text{lncRNA}}^{2}\right)}. \end{array}$$

The key lncRNAs in LUAD were identified using the above formula, and the coefficients of each key lncRNAs were computed via the univariable Cox proportion risk model, and the equation to compute the risk scoring for every sufferer was stated below: Score = ∑*β* *i* × Expi. Herein, *i* represents the expressions of glutamine metabolism-related lncRNAs, and *β* refers to the coefficient of the corresponding lncRNA acquired from the univariate Cox model. Sufferers were classified into high-risk group and low-risk group on the foundation of the median expression. The K-M method was used to finish survival analyses, and the statistic differences in survival between these two groups were analyzed using the log-rank test.

The article "Comprehensive Analysis of Subtypes and Identification of Key lncRNAs Based on Glutamine Metabolism-Related Long Noncoding RNAs" was retracted in 2023. Reasons: signs of a paper mill; compromised peer review; unreliable results or conclusions.

### 2.10. Statistical Analysis

The entire statistic assay was completed via the R program (version 4.0.3). Comparisons between three or more groups were made via the Kruskal-Wallis test. *P* < 0.05 had significance on statistics.

## 3. Results

### 3.1. Identification of Three LUAD Molecular Subtypes according to Glutamine Metabolism-Related Scores

First, by correlation analysis of glutamine metabolism score with lncRNA expression, 2207 (14.9%), 157 (4.7%), and 251 (4.8%) glutamine metabolism-related lncRNAs were identified in TCGA-LUAD, GSE31210, and GSE72094 cohorts, respectively. A total of 11 glutamine metabolism-related lncRNAs were shared commonly among the three cohorts (Figure 1(a)), which suggested that glutamine metabolism-related lncRNAs were less consistently expressed between datasets from different platforms. Thus, the 11 lncRNAs were selected for subsequent analysis. The CDF and the relative change in the area under the CDF curve showed no significant increase with increasing *k* beyond *k* = 3 (Figures 1(b) and 1(c)). Therefore, LUAD samples were divided into three molecular subtypes (Figure 1(d)). K-M curves revealed that the OS of sufferers with LUAD became increasingly longer from cluster 1 (C1) to cluster 3 (C3) in TCGA-LUAD, GSE31210, and GSE72094 cohorts (Figures 1(e)–1(g)). There were significant differences in glutamine scores among the three subtypes in the three datasets, with progressively lowered glutamine scores from cluster 1 (C1) to cluster 3 (C3) (Figures 1(h)–1(j)).

### 3.2. Genomic Alterations in Three Glutamine Metabolizing Subtypes

We investigated the genomic alterations in three glutamine metabolizing subtypes. In the TCGA dataset, the aneuploidy score, HRDs, fraction altered, number of segments, and TMB were significantly different among the three glutamine metabolizing subtypes. The aneuploidy score, HRDs, fraction altered, number of segments, and tumor mutational burden (TMB) were always higher for C1 relative to C2 and C3 (Figure 2(a)). In particular, aneuploidy score, HRDs, fraction altered, and number of segments were all significantly positively correlated with glutamine metabolism score (Figure 2(b)). The top 10 genes with mutations, copy number deletions, and amplification frequencies in the three subtypes are shown in Figure 2(c). Based on the results from the waterfall plot, STK11 (39%), Kelch-like ECH associated protein 1 (KEAP1) (35%), ATM (28%), and Helicase For Meiosis 1 (HFM1) (22%) had the highest mutation rates in C1; in particular, mutation rates for TK11 and KEAP1 in C1 even exceeded the sum of mutation rates in C2 and C3. In addition, the incidence of both copy number amplification and deletion of genes were significantly higher in C1 relative to C2 and C3 (Figure 2(c)). Thus, the genome of C1 was the most unstable among the three subtypes.

The article "Comprehensive Analysis of Subtypes and Identification of Key lncRNAs Based on Glutamine Metabolism-Related Long Noncoding RNAs" was retracted in 2023. Reasons: signs of a paper mill; compromised peer review; unreliable results or conclusions.

### 3.3. Analysis of the Regulatory Pathways of Glutamine Metabolic Subtypes

To compare regulatory pathways among the glutamine metabolizing subtypes, GSEA was performed, and 16 pathways were found to be significantly inhibited in the C1 subtype relative to C3 of the TCGA-LUAD dataset. Three and 16 significantly inhibited pathways were identified in the C1 subtype of the GSE31210 and GSE72094 cohorts, respectively. The significantly inhibited pathways detected in all three datasets included myogenesis, TNF-*α* signaling via NF-*κ*B, and allograft rejection (Figure 3(a)). We selected the pathways in the C1 subtype that were inhibited in both TCGA-LUAD and GSE72094 cohorts and attempted to compare the differences in the status of these pathways between C1 and C2 and between C2 and C3 subtypes by plotting radar plots and estimating the normalized enrichment scores (NESs) of GSE31210 between C1 and C2 and between C2 and C3 subtypes. Multiple pathways that regulate tumor immunity, including IFN*α* response, allograft rejection, inflammation response, complement activation, and interferon-gamma response, were significantly downregulated in C1. In addition, these tumor immune-related pathways were markedly activated in C3 compared to C2 (Figures 3(b)–3(d)). Thus, C1 had the weakest antitumor immunity and C3 the strongest; C2 had intermediate values.

### 3.4. TME of Glutamine Metabolic Subtypes

Given the differential antitumor immunity among the glutamine subtypes, our team further studied the distribution of immunocytes in the TME of the three glutamine metabolizing subtypes. Immune cells within TME in TCGA-LUAD, GSE31210, and GSE72094 cohorts were first analyzed using the ssGSEA algorithm. Relative to the other two glutamine metabolizing subtypes, C1 showed immune cell underinfiltration. The TME of C2 was enriched with a large proportion of immunosuppressive cells, such as dendritic cells, NK cells, Th1 cells, and Treg cells. The TME of C3 showed the highest infiltration of leukocytes (eosinophils, neutrophils) (Figures 4(a)–4(c)). In all three datasets, the immune and stromal scores of C1 were significantly lower than those in C2 and C3 subtypes (Figures 4(d)–4(f)). Next, unsupervised hierarchical clustering based on C1 and C3 immune cell scores categorized the specimens in the three cohorts into high- and low-immune infiltration groups. Most C1 samples were clustered in the low immune infiltration group, while C3 samples pooled together in the high immune infiltration group. Along with the results as shown in Figure 3, we inferred that C1 may be an immunodeficient phenotype, C2 an immunosuppressive phenotype, and C3 an immune-activating phenotype.

The article "Comprehensive Analysis of Subtypes and Identification of Key lncRNAs Based on Glutamine Metabolism-Related Long Noncoding RNAs" was retracted in 2023. Reasons: signs of a paper mill; compromised peer review; unreliable results or conclusions.

### 3.5. Immunotherapeutic Responses of Glutamine Metabolizing Subtypes

We also examined the responses to immunotherapy among the glutamine metabolizing subtypes. First, the immune checkpoint expression of glutamine subtypes in the three cohorts was compared. The results showed that almost all of the 21 immune checkpoints were differentially expressed between C1 and C3, wherein the C1 subtype showed the least expression (Figure S2). Specifically, 20 of the 21 immune checkpoints were differentially expressed among the three subtypes in TCGA-LUAD, and 19 and 18 were differentially expressed among the glutamine metabolizing subtypes in the GSE31210 and GSE72094 cohorts, respectively (Figures 5(a)–5(c)). Moreover, our team combined the frequency of immune checkpoint abnormalities among patients with different glutamine subtypes in the three cohorts (Figure 5(d)). Next, the TIDE scores for different glutamine metabolism subtypes were evaluated, and no significant differences were found in TCGA dataset; however, the TIDE score of the C3 subtype was the lowest. The effects of immunotherapy predicted using the TIDE software in different glutamine metabolizing subtypes of TCGA-LUAD were analyzed, and the outcomes revealed that the C3 subtype exhibited the highest response rate to immunotherapy relative to the other two glutamine metabolizing subtypes (Figure 5(e)). In the GSE31210 cohort, the TIDE scores were significantly different among the glutamine metabolizing subtypes. The C2 and C3 subtypes were significantly more likely to benefit from immunotherapy than C1 (Figure 5(f)). These results were consistent in the GSE72094 cohort (Figure 5(g)). Thus, the C3 subtype was more sensitive to immunotherapy.

The article "Comprehensive Analysis of Subtypes and Identification of Key lncRNAs Based on Glutamine Metabolism-Related Long Noncoding RNAs" was retracted in 2023. Reasons: signs of a paper mill; compromised peer review; unreliable results or conclusions.

### 3.6. Localization and Transcriptional Regulatory Mechanisms of Glutamine Metabolism-Associated lncRNAs

We compared the relationship between glutamine metabolism-associated lncRNAs and protein-coding genes with glutamine metabolic activity, and the correlation coefficient density curves showed that the glutamine metabolism-associated lncRNAs were negatively associated with glutamine metabolic activity relative to the glutamine metabolism-associated protein-coding genes (PCGs) in the three LUAD datasets (Figure 6(a)). The subcellular localization of lncRNAs determines their mode of action. Thus, we investigated the mode of action of glutamine metabolism-associated lncRNAs by predicting the localization of the 11-glutamine metabolism-related lncRNAs using the LncATLAS database. The pie chart demonstrates the proportions (%) of lncRNAs with positive or negative values in the RCI. The results indicated that the majority of glutamine metabolism-related lncRNAs were localized to the nucleus (Figure 6(b)). Binding to the TFs to modulate genetic transcription is the primary mechanism of action for the lncRNAs in the nucleus [25]. We therefore further investigated the association of shared glutamine metabolism-related lncRNAs in the three cohorts with TFs, and as shown in Figure 6(c), a set of TFs was significantly negatively associated with glutamine metabolism-related lncRNAs. Based on the degree of correlation of the 11 lncRNAs with TFs, we selected nine among them for predicting the subcellular localization (Figure 6(d)). Through the differential analysis of TF activation for the three glutamine metabolism subtypes in each LUAD study cohort, 49 TFs in TCGA-LUAD and 39 and 43 TFs in the GSE31210 and GSE72094 cohorts, respectively, were identified. Nine of these upregulated TFs were common among the three LUAD datasets, namely, MYC, E2F4, E2F1, YY1, AR, CCCTC-binding factor (CTCF), forkhead box protein M1 (FOXM1), nuclear factor I C (NFIC), and forkhead box protein P1 (FOXP1) (Figure 6(g), Figure S3). The expressions of these TFs were significantly negatively correlated with the expression of glutamine metabolism-associated lncRNAs (Figure 6(h)). We counted the number of activated and suppressed TFs in C1 relative to C3 in the three LUAD cohorts (Figure 6(e)). The biological pathways of TF enrichment were analyzed, and these TFs were significantly associated with infection and the cell cycle of viruses causing human cancer (Figure 6(f)). Thus, glutamine metabolism-related lncRNAs may likely be involved in cancer progression through the TFs.

The article "Comprehensive Analysis of Subtypes and Identification of Key lncRNAs Based on Glutamine Metabolism-Related Long Noncoding RNAs" was retracted in 2023. Reasons: signs of a paper mill; compromised peer review; unreliable results or conclusions.

### 3.7. Identification of Glutamine Metabolism-Associated lncRNAs That Predict Prognosis of LUAD

Finally, to identify the key lncRNAs from among the glutamine metabolism-related lncRNAs, a first-order bias correlation analysis was performed. The glutamine metabolism scores and glutamine metabolism-related genes showed that the adjustment of nine glutamine metabolism-related lncRNAs could alter the correlation coefficients of glutamine metabolism-related genes. Among them, the correlation between glutamine metabolism score and glutamine metabolism-related genes was significantly weakened after removing the effects of three lncRNAs (MAGI2-AS3, NR2F1-AS1, and LINC00921) (Figure 7(a)). Genes that were significantly negatively correlated with the three lncRNAs were significantly enriched in the ribosome, biosynthesis of amino acids, carbon metabolism, citrate cycle (TCA cycle), 2-oxocarboxylic acid metabolism, and other metabolic pathways (Figure 7(b)). Risk models based on MAGI2-AS3, NR2F1-AS1, and LINC00921 allowed for scoring the risk in each patient in TCGA-LUAD, GSE31210, and GSE72094 datasets; the patients with LUAD having a low-risk score had significantly longer OS relative to those with a high-risk score (Figure 7(c)). In addition, we also observed the expression differences of MAGI2-AS3, NR2F1-AS1, and LINC00921 in different subtypes. It can be observed that the expression of three lncRNAs is significantly low in C1 subtype, and MAGI2-AS3 and NR2F1-AS1 are significantly high in C2 subtype (Figure S4A). It is worth mentioning that the expression of MAGI2-AS3 is highly positively correlated with multiple immune infiltrating cells, while NR2F1-AS1 and LINC00921 are significantly negatively correlated with multiple immune infiltrating cells (Figure S4B). Comparing the relationship between the expression of these three lncRNAs and the characteristics of genomic variation, it can be observed that there are significant differences in animal, homologous recombination defects, fraction altered, number of segments, and tumor mutation burden in the samples with high and low expression of MAGI2-AS3. The high expression of MAGI2-AS3 is related to the high genomic variation (Figure S5). These results suggest that MAGI2-AS3, NR2F1-AS1, and LINC00921 are important potential molecular markers in lung adenocarcinoma.

## 4. Discussion

Previous evidence strongly suggests that lung cancer is a metabolic disorder. The metabolic and energy production networks in lung cancer cells are rewired to support their survival and rapid proliferation [26]. Frequent alterations in glucose metabolism in oncocytes have been used for the diagnoses and therapies of cancer. The roles of other glycolysis intermediates, alternative pathways for energy production, and macromolecule synthesis in oncocytes have been acknowledged very recently. In particular, the crucial effects of varied glutamine metabolism underlying the malignant behaviors of oncocytes and the possible therapeutic utility of such cell adaptation have become an essential investigation hotspot in the field of cancer biology [27]. Some studies in recent years also hint at the vital roles of lncRNAs in glutamine metabolism; nevertheless, our knowledge of lncRNAs in glutamine metabolism in tumors remains limited as compared to that of PCGs in the regulation of metabolism in cancer [28].

The article "Comprehensive Analysis of Subtypes and Identification of Key lncRNAs Based on Glutamine Metabolism-Related Long Noncoding RNAs" was retracted in 2023. Reasons: signs of a paper mill; compromised peer review; unreliable results or conclusions.

We Given the increased expression levels of glutamine in the pulmonary carcinoma tissues relative to other cancer types, particularly in NSCLC, relative to other carcinoma types (e.g., colon carcinoma or gastric carcinoma) [29]. Herein, our team explored the glutamine metabolism-associated lncRNAs in the LUAD subtype of NSCLC. We identified 11 commonly shared glutamine metabolism-related lncRNAs in three different LUAD data cohorts using glutamine metabolism scores and ssGSEA. Several previous studies have highlighted the metabolic heterogeneity in lung tumors [30], suggesting that LUAD may have different metabolic phenotypes. To investigate the metabolic phenotypes, we classified the LUAD samples into three glutamine metabolic subtypes based on the 11 glutamine metabolism-associated lncRNAs. Among these, the C1 subtype was found to be the most unstable. An earlier study by Mariam Jamal-Hanjani et al. shows that this feature of the chromosome is related to an increased risk of relapse or death. We found that the risk of death in C1 was indeed the highest among the three glutamine metabolic subtypes.

Glutamine metabolism not only promotes cancer growth but creates an immunosuppressive microenvironment. The blockade of glutamine metabolism can disturb the entire tumor metabolism and significantly enhance endogenous antitumor immunity [31]. Herein, we found that multiple immunomodulatory pathways in C1, including inflammation response, IFN*α* response, IFN-*γ* response, allograft rejection, and complement activation, were among the most downregulated; the immune score of C1 was the lowest, and the infiltration of immune cell types in the TME was insufficient. The TME of C2 was enriched with a large number of immunosuppressive cells, such as the dendritic cells, NK cells, Th1 cells, and Treg cells. The tumor immunoregulatory pathways were activated in C3, and the infiltration of leukocytes in the TME was the highest. In addition, unsupervised hierarchical clustering based on immune cell scores for C1 and C3 also showed that most of the C1 samples were clustered in the low immune infiltration group, while those of C3 were pooled in the high immune infiltration group. Thus, we speculated that C1 may be an immunodeficient phenotype, C2 an immunosuppressive phenotype, and C3 an immune-activating phenotype.

The article "Comprehensive Analysis of Subtypes and Identification of Key lncRNAs Based on Glutamine Metabolism-Related Long Noncoding RNAs" was retracted in 2023. Reasons: signs of a paper mill; compromised peer review; unreliable results or conclusions.

To comprehensively understand their biology, the cumulative evidence involving lncRNA in almost every cellular activity renders the assessment of their subcellular localization cardinal [32]. Several lncRNAs are located in nuclei, either enriched in chromatin or located in specific subnucleus compartments. Nuclear lncRNAs are involved in some biology processes, such as chromatin organization, transcription, and posttranscriptional genetic expression. They also serve as structure scaffolds for nuclear domains [33]. For the 11-glutamine metabolism-associated lncRNAs, our analysis showed their predominant localization in the nucleus. Nine potential TFs associated with these lncRNAs, which were significantly associated with infection and the cell cycle of viruses that cause human cancer, were also predicted. We hypothesized that glutamine metabolism-related lncRNAs may likely interact with TFs to regulate the biological processes in LUAD.

Finally, by first-order partial correlation analysis, we identified three lncRNAs, enriched in multiple metabolic pathways. Most of these lncRNAs are related to tumor invasion and metastasis. MAGI2-AS3 is generally expressed in human cancer. The expression level of MAGI2-AS3 is related to cancer progression and prognosis. The imbalance of MAGI2-AS3 regulates cancer cell proliferation, cell death, and metastasis by acting as competitive endogenous RNA (ceRNA), epigenome regulator, and transcription regulator invasion, metastasis, and treatment resistance [34]. Previously, Song et al. [35] reported that in non-small-cell lung cancer, MAGI2-AS3 is related to radiation response and effectively predicts the prognosis of patients. As a tumor suppressor, MAGI2-AS3 weakens the progression of non-small-cell lung cancer by targeting the mir-629-5p/TXNIP axis [36]. NR2F1-AS1 expression is upregulated in non-small-cell lung cancer cells (NSCLC), which is associated with adverse clinical features and short overall survival in NSCLC patients. The deletion of NR2F1-AS1 functionally reduces the proliferation, migration, and invasion of NSCLC cells and promotes tumor cell apoptosis [37]. Only a few studies have reported the regulatory mechanisms of these three lncRNAs localized in the nucleus in cancer metabolism. Therefore, in the future, we intend to investigate the mechanisms of MAGI2-AS3, NR2F1-AS1, and LINC00921 in LUAD metabolism using experiments in vitro cell assay and in vivo tumor assay.

The article "Comprehensive Analysis of Subtypes and Identification of Key lncRNAs Based on Glutamine Metabolism-Related Long Noncoding RNAs" was retracted in 2023. Reasons: signs of a paper mill; compromised peer review; unreliable results or conclusions.

## 5. Conclusion

In summary, we identified three LUAD subgroups classified according to the glutamine metabolism-associated lncRNAs that exhibited distinct genomic profiles, TME profiles, and sensitivity to immunotherapy. We inferred that C1 represented an immunodeficient phenotype, C2 an immunosuppressive phenotype, and C3 an immune-activating phenotype in each glutamine metabolism subgroup. Finally, three key glutamine metabolism-associated lncRNAs were screened. This investigation provided new findings for the development of new and valid treatment regimens that target tumorous metabolic pathways.

## Figures and Tables

**Figure 1:** Identification of molecular subtypes of LUAD based on glutamine metabolism scores. (a) Venn diagram of shared glutamine metabolism-related lncRNAs in TCGA-LUAD, GSE31210, and GSE72094 cohorts. (b) CDF curve for TCGA-LUAD. (c) Relative change of the area under the CDF curve for TCGA-LUAD. (d) Consensus matrix for TCGA-LUAD at *k* = 3. (e–g) Kaplan-Meier curves for patient survival in the TCGA-LUAD, GSE31210, and GSE72094 datasets. (h–j) Glutamine metabolism scores for the three molecular subtypes in TCGA-LUAD, GSE31210, and GSE72094 cohorts. *P* values are marked with ^∗^ above each violin plot; ^∗^*P* < 0.05; ^∗∗^*P* < 0.01; ^∗∗∗^*P* < 0.001; ^∗∗∗∗^*P* < 0.0001.

**Figure 2:** Genomic differences in the three glutamine metabolizing subtypes. (a) Aneuploidy score, HRDs, fraction altered, number of segments, and TMB for each glutamine metabolizing subtype from left to right. (b) Pearson correlation analysis for glutamine metabolizing score with aneuploidy score, HRDs, fraction altered, number of segments, and TMB. (c) Mutations, copy number deletions, and amplification frequencies for the top 10 genes in C1-C3 from left to right. *P* values are marked with ^∗^ above each violin plot; ^∗^*P* < 0.05; ^∗∗^*P* < 0.01; ^∗∗∗^*P* < 0.001; ^∗∗∗∗^*P* < 0.0001.

**Figure 3:** Analysis of regulatory pathways in glutamine metabolic subtypes. (a) The thermal graph displaying NESs of Hallmark pathways computed on comparison of C1 and C3 subtypes. (b, c) Radar plots showing NESs of Hallmark pathways computed using GSEA of C1 versus C2 and C2 versus C3 in TCGA and GSE72094 cohorts. (d) Performance of NESs between C1 and C2 and between C2 and C3 for samples in the GSE31210 cohort.

**Figure 4:** TME of glutamine metabolic subtypes. (a–c) ssGSEA scores of glutamine metabolizing subtypes for TME in TCGA-LUAD, GSE31210, and GSE72094 cohorts in different components. (d–f) Immune score, stromal score, and ESTIMATE score of glutamine metabolizing subtypes in TCGA-LUAD, GSE31210, and GSE72094. (g–i) Unsupervised hierarchical clustering of samples into high- and low-immune infiltration groups based on immune cell scores for C1 and C3 in TCGA-LUAD, GSE31210, and GSE72094 cohorts. *P* values are marked with ^∗^ above each box plot; ^∗^*P* < 0.05; ^∗∗^*P* < 0.01; ^∗∗∗^*P* < 0.001; ^∗∗∗∗^*P* < 0.0001.

The article "Comprehensive Analysis of Subtypes and Identification of Key lncRNAs Based on Glutamine Metabolism-Related Long Noncoding RNAs" was retracted in 2023. Reasons: signs of a paper mill; compromised peer review; unreliable results or conclusions.

**Figure 5:** Immunotherapeutic responses of glutamine metabolizing subtypes. Analysis of differential expression for the 21 immune checkpoints among the three glutamine metabolic subtypes in TCGA-LUAD (a), GSE31210 (b), and GSE72094 (c). (d) The bar plot indicates frequencies of abnormal immune checkpoints among subtypes of cancer patients across the three cohorts. The *x* axis represents the number of cohorts, and the *y*-axis shows the names of immune checkpoints. The effects of immunotherapy predicted among the different glutamine metabolism subtypes using the TIDE software in the TCGA-LUAD (e), GSE31210 (f), and GSE72094 (g) cohorts. ^∗^ represents *P* < 0.05, ^∗∗^ represents *P* < 0.01, ^∗∗∗^ represents *P* < 0.0001, and ns represents no significant difference.

**Figure 6:** Localization and regulatory transcriptional mechanisms underlying glutamine metabolism-related lncRNAs. (a) Density curves for correlation coefficients of glutamine metabolism-associated lncRNAs and protein-coding genes (PCGs). (b) Percentages of lncRNAs with negative or positive values in the relative concentration index (RCI). (c) Frequencies of TFs associated with glutamine metabolism-associated lncRNAs. (d) Subcellular localization of the nine lncRNAs. (e) Number of suppressed or activated TFs in C1 relative to C3 in the three LUAD cohorts. (f) Enriched biological pathways involving the TFs. (g) Expression of nine upregulated TFs common among the glutamine metabolizing subtypes in the three LUAD datasets. (h) Correlation of TF expression with that of glutamine metabolism-associated lncRNAs. ^∗^*P* < 0.05; ^∗∗^*P* < 0.01; ^∗∗∗^*P* < 0.001; ^∗∗∗∗^*P* < 0.0001.

**Figure 7:** Identification of key glutamine metabolism-related lncRNAs and their functions in LUAD. (a) Cumulative distribution curve (CDF) of glutamine metabolism-related genes in the presence or absence of adjustment for lncRNAs via the first-order partial correlation analysis. The *x*-axis denotes the Pearson correlation coefficient between glutamine metabolism score and genetic expression, and the *y*-axis indicates the cumulative probability. The solid line represents the CDFs of glutamine metabolism scores and gene expression correlation coefficients before adjustment, and the dashed line represents the CDFs of glutamine metabolism scores and gene expression correlation coefficients adjusted using the first-order partial correlation analysis. (b) Bubble plots for pathway enrichment of genes significantly negatively correlated with the expression of MAGI2-AS3, NR2F1-AS1, and LINC00921. (c–e) Survival curves of patients having different risks in TCGA-LUAD, GSE31210, and GSE72094 datasets.

The article "Comprehensive Analysis of Subtypes and Identification of Key lncRNAs Based on Glutamine Metabolism-Related Long Noncoding RNAs" was retracted in 2023. Reasons: signs of a paper mill; compromised peer review; unreliable results or conclusions.

## Data Availability

The data used to support the findings of this study are included within the article.

## Supplementary Materials

Supplementary Materials Figure S1: work flow chart. Figure S2: analysis of differential expression of 21 immune checkpoints among glutamine metabolic subtypes in TCGA-LUAD, GSE31210, and GSE72094 datasets. Figure S3: expressions of nine upregulated TFs among glutamine metabolizing subtypes in the GSE31210 and GSE72094 cohorts. Figure S4: expression relationship of three lncRNAs. (A) The expression and distribution of the three lncRNAs in the three molecular subtypes were different. (B) Correlation between the expression of three lncRNAs and immune infiltrating cells. Figure S5: relationship between the expression of three lncRNAs and genomic variation.
